The article "Phyllanthus reticulatus Prevents Ethanol-Induced Gastric Ulcer via Downregulation of IL-8 and TNF-α Levels" was published in 2021. Journal: Evid Based Complement Alternat Med.

# *Phyllanthus reticulatus* Prevents Ethanol-Induced Gastric Ulcer via Downregulation of IL-8 and TNF-*α* Levels

**DOI:** 10.1155/2021/1734752

**Published:** 2021-09-24

**Authors:** Hafsa Izhar, Arham Shabbir, Muhammad Shahzad, Aisha Mobashar, Syed Shoaib Ahmed

**Affiliations:** ^1^Department of Pharmacology, Faculty of Pharmacy, The University of Lahore, Lahore Campus, Lahore, Pakistan; ^2^Institute of Pharmacy, Faculty of Pharmaceutical and Allied Health Sciences, Lahore College for Women University, Jail Road, Lahore, Pakistan; ^3^Department of Pharmacology, University of Health Sciences, Lahore, Punjab, Pakistan; ^4^Centre for Research in Molecular Medicine, The University of Lahore, Lahore Campus, Lahore, Pakistan

## Abstract

The current study aimed to determine the protective effect of *P. reticulatus* on ethanol-induced gastric ulcer. For this purpose, thirty-six Sprague-Dawley rats were divided into six groups. The first group served as normal control, while, in other five groups, absolute ethanol was used to induce gastric ulcer. Group II served as a diseased group, while groups III, IV, and V were treated with methanol extract, ethyl acetate fraction, and *n*-hexane fraction, respectively, in a dose of 400 mg/kg bodyweight. Group VI was given omeprazole in a dose 20 mg/kg bodyweight. The stomachs were removed, ulcer score was evaluated, and histopathological examination of gastric lumen was conducted. Total acidity and pH values were determined in gastric juice. TNF-*α* and IL-8 mRNA expressions levels were determined using the reverse transcription real-time PCR method. The data indicated that *P. reticulatus* protected against gastric ulcer, which was evident by attenuation of ulcer score. The pretreatment with *P. reticulatus* raised the gastric pH and improved all evaluated histopathological parameters such as ulcer score, erosion score, hemorrhage score, fibrinoid necrosis score, inflammatory infiltrate score, and edema score. *P. reticulatus* significantly reduced mRNA expression levels of TNF-*α* and IL-8. In conclusion, *P. reticulatus* possess antiulcer property which might be attributed to downregulation of TNF-*α* and IL-8 expression levels.

## 1. Introduction

The pathophysiology of peptic ulcers is mainly focused between aggressive (chloride corrosive effects and pepsin) and defensive elements (body fluids, bicarbonate secretions, prostaglandins, sulfhydryl compounds, polyamines, nitric oxide, and dopamine) [1]. Abdominal pain, epigastric tenderness, nausea, ample vomiting, and distention are common signs and symptoms [2]. Microscopic appearance determines the base of the ulcer in 4 zones, i.e., inflammatory exudate, fibrinoid necrosis, tissue granulation, and fibrous tissue during the active stage. The fibrous base of the ulcer may contain vessels with thickened wall or with thrombosis [3].

The article "Phyllanthus reticulatus Prevents Ethanol-Induced Gastric Ulcer via Downregulation of IL-8 and TNF-α Levels" was published in 2021. Journal: Evid Based Complement Alternat Med.

Therapeutic management and treatment of peptic ulcer includes several classes of drugs, i.e., (PPI's) proton pump inhibitors, histamine receptor blockers, mucosal blockers, and prostaglandin analogs. However, development of tolerance and side effects has led to doubts about the efficacy of these drugs, suggesting the need to develop new drugs against ulcers [4]. Plant-derived medicinal treatment is common and extends to traditional and modern medicinal practice. As stated by the World Health Organization, more than 80% of community in developing countries is largely dependent on herbal medicine [5].

*Phyllanthus reticulatus* Poir. (family: Euphorbiaceae), commonly known as pancoli or carinelli, is a giant hairless or pubescent shrub with smooth or lenticular late branches, 8–10 feet in height. Its leaves are oval to elliptical or obovate, and the organic product is purple dark berries [6]. The plant is known to have analgesic, anti-inflammatory, cholesterol lowering, cytotoxic, immunomodulatory, antidiabetic, antimalarial, antibacterial, and hepatoprotective effects [7]. In the traditional system of medicine, the plant is used as a remedy of gastrointestinal disorders [8]. The ethanol-induced gastric ulcer model is widely used to evaluate the gastric cytoprotective effect of plant extract against ingested irritants. The current study aimed to evaluate the immunomodulatory activities of *P. reticulatus* against ingested irritants using ethanol-induced gastric ulcer model in rats.

## 2. Methodology

### 2.1. Plant Collection

*Phyllanthus reticulatus* was collected from the botanical garden of Government College University, Lahore, and the specimen was confirmed by Dr. Zaheer-u-din at the Department of Botany, Government College University, Lahore. A specimen voucher was deposited in the herbarium of the University (GC.Herb.Bot.3474).

### 2.2. Preparation of the Plant Extract and Fractionation

The collected plant leaves were carefully washed to remove contaminants. The leaves were dried in the air under shadow for 15 days and powdered using the grinder. The ground powder (500 g) was immersed in 2 liters of methanol using an airtight glass bottle. The bottle was stored at room temperature for 7 days with recurrent shaking. The material was first filtered with muslin cloth and then by using filter paper (Whatman number 1).

The obtained filtrate was evaporated by using the rotary evaporator under low pressure to obtain semisolid thick extract. Then, the crude methanolic extract was dissolved in 200 ml distilled water.

The article "Phyllanthus reticulatus Prevents Ethanol-Induced Gastric Ulcer via Downregulation of IL-8 and TNF-α Levels" was published in 2021. Journal: Evid Based Complement Alternat Med.

The obtained solution was placed for liquid-liquid extraction, by using *n*-hexane and separating funnel. The *n*-hexane fraction was collected, and the excessive solvent was evaporated using the rotary evaporator under low pressure. After separating the *n*-hexane layer, the aqueous layer was again subjected to fractionation by using ethyl acetate solvent [9].

### 2.3. Experimental Animals

Thirty-six Sprague-Dawley rats, 150–250 grams, of either sex, were divided into six groups each having 6 rats. Animals were maintained in the animal house of the University of Lahore at controlled room temperature (26 ± 2°C) and humidity (40–60%) conditions. Dark and light cycles (12 hours) were also ensured. Rats were fed on standard diet and water ad libitum [10]. The experiments were approved by Institutional Research Ethics Committee, the University of Lahore (IREC-2018-52).

### 2.4. Experimental Design

#### 2.4.1. Group І (Naive)

Normal saline was given to rats in this group.

#### 2.4.2. Group II (Vehicle Control)

Ethanol was given orally to rats at a dose of 5 ml/kg b.w. in a single dose by the gavage method [11].

#### 2.4.3. Group III (Meth-Treated)

Methanolic extract of *P. reticulatus* was given at a dose of 400 mg/kg b.w., p.o. [12]. Then, after 1 h of extract administration, ethanol (100%) was given in a single oral dose (5 ml/kg b.w.).

#### 2.4.4. Group IV (NH-Treated)

Rats were pretreated with *n*-hexane fraction of *P. reticulatus* at a dose of 400 mg/kg b.w., p.o. [12]. Then, after 1 h of pretreatment, absolute ethanol was administered in a single oral dose (5 ml/kg b.w.).

#### 2.4.5. Group V (EA-Treated)

This group was pretreated with ethyl acetate fraction of *P. reticulatus* at a dose of 400 mg/kg b.w., p.o. [12]. Absolute ethanol was administered (5 ml/kg b.w.) after 1 h of pretreatment with ethyl acetate fraction.

#### 2.4.6. Group VI (OM-Treated)

Omeprazole was given to rats in this group at a dose of 20 mg/kg b.w., p.o. [13]. Subsequently, absolute ethanol was administered (5 ml/kg b.w.) after 1 h of pretreatment.

### 2.5. Pylorus Ligature and Removal of Gastric Tissue

Rats were sacrificed after two hours of ethanol administration [14]. The stomachs were first ligated with thread from both ends. The stomachs were punctured through sterilized needle, and gastric juice was collected within Eppendorf tubes [15]. Then, stomachs were opened along greater curvature for two parameters. One sample was immersed in 10% buffered formalin for histopathological analysis and kept at room temperature. Another sample was immersed in 100 ml TRIzol reagent for RT-PCR analysis and kept at -80 °C.

### 2.6. Ulcer Score

Morphological features of the gastric ulcer such as redness, erythema, and hemorrhage were determined. Ulcer score was measured by giving 0 to normal mucosa/no ulcer, 1 to mucosal lesion limited to superficial layer/superficial ulcer, 2 to mucosal lesion penetrated to deep layer/deep ulcer, and 3 to mucosal damage with a hole/perforation [16].

The article "Phyllanthus reticulatus Prevents Ethanol-Induced Gastric Ulcer via Downregulation of IL-8 and TNF-α Levels" was published in 2021. Journal: Evid Based Complement Alternat Med.

### 2.7. Determination of Gastric Acidity and pH

The stomachs were removed, and gastric contents were collected to measure pH values. The gastric contents were centrifuged at 1200 rpm for 10 minutes, and pH values were determined. Total acid in gastric juice was evaluated in supernatant by titration as pH 7.0 with 0.01 N NaOH solution and phenolphthalein as an indicator [17].

### 2.8. Histopathological Assessment

For histopathological examinations, stomach tissues were immersed in 10% buffered formalin, fixed in formalin solution. After fixation, the stomachs were cut open longitudinally along greater curvature, and pathological changes in the stomach lumen were observed. 2-3 mm thick sections from representative areas were taken and processed to prepare paraffin blocks. Section was cut at 5 *µ*m of thickness and stained with hematoxylin and eosin [18]. Sections were then evaluated microscopically for histological changes including erosions, edema, hemorrhage, fibrinoid necrosis, and inflammatory cell infiltration.

### 2.9. Evaluation of mRNA Expression Levels of IL-8 and TNF-*α* using qRT-PCR Analysis

#### 2.9.1. Extraction of RNA and Synthesis of Complementary DNA

Briefly, gastric tissues were mixed with TRIzol reagent and homogenized. 150 *µ*L of chloroform were added, contents were centrifuged, and the top transparent layer (aqueous phase) containing RNA was separated. Then, isopropanol of equal proportion was added for precipitation of RNA. The RNA pellets were washed with 1 ml of 75% ethanol. RNase free water (20 *µ*L) was added to solubilize RNA pellet. The quantity of RNA was measured using the nanodrop spectrophotometer.

cDNA was synthesized by reverse transcription using the cDNA synthesis kit (Thermo scientific America). 1000 ng of RNA from each sample was mixed with oligo dt primer (10 *µ*M), nuclease free water, centrifuged, placed in the thermal cycler for heating for 5 min at 70^o^C, and immediately chilled afterwards. Further components of the kit were added, i.e., 4 *µ*L of 5X reaction buffer, 0.5 *µ*L of RNase inhibitor (20 U/*µ*L), 2 *µ*L of dNTP mix (10 mM), and 0.5 *µ*L of MMuLV enzyme (200 U/*µ*L). All PCR tubes were placed in the thermal cycler (BioRad, USA) for 60 min at 40°C [19].

### 2.10. Real-Time Polymerase Chain Reaction (qPCR)

For amplification, 2 *µ*L of cDNA was mixed with 1.5 *µ*L of reverse and forward primer, each (10 *µ*M), 6 *µ*L of PCR Master Mix containing SYBR green dye, and 2 *µ*L of nuclease free water q.s. to 12 *µ*l. Thermal cycler was programed for denaturation cycle at 95^o^C for 10s, annealing at 60^o^C for 30s (cycles = 45), and extension at 72^o^C for 30s. Gene expression levels were recorded as threshold cycle (Ct) values.

The article "Phyllanthus reticulatus Prevents Ethanol-Induced Gastric Ulcer via Downregulation of IL-8 and TNF-α Levels" was published in 2021. Journal: Evid Based Complement Alternat Med.

### 2.11. Statistical Analysis

Data were analyzed using GraphPad Prism v.6 software and presented in the form of mean ± standard deviation. To analyze quantitative variables, one-way ANOVA was used. To compare all groups with each other, the post hoc Tukey's test was used.

## 3. Results

### 3.1. Histopathological Studies

Pretreatment with plant extracts and omeprazole attenuated ulcer score, erosion score, hemorrhage erosion, fibrinoid score, inflammatory infiltrate score, and edema score (Figure 1; Table 1).

### 3.2. Measurement of Gastric pH

Gastric contents of each rat were collected and centrifuged at 3000 rpm for 10 min. Graphical representation shows the pH changes in the diseased group and treated groups after ulcer induction with ethanol. Significantly lower pH was observed in the vehicle control group rats as compared with the naive group (5.400 ± 0.3521 vs. 6.950 ± 0.4324). The pH values were found significantly (*P* < 0.001) increased in the Meth-treated group (7.350 ± 0.2881), EA-treated group (7.383 ± 0.1941), NH-treated group (7.300 ± 0.1789), and OM-treated group (7.400 ± 0.1897) (Figure 2).

### 3.3. Measurement of Total Gastric Acidity

Total gastric acidity was measured from the gastric contents of normal, diseased, and treated groups of rats. It was found that the total acidity was substantially decreased (*P* < 0.001) in OM-treated (57.2 ± 1.82), NH-treated (61.3 ± 2.42), EA-treated (61.8 ± 1.62), and Meth-treated groups (62.3 ± 1.61) in comparison to the vehicle control group (76.3 ± 2.79) (Figure 3).

### 3.4. Effects of *P. reticulatus* on Ulcer Score

Results showed elevated (*P* < 0.001) ulcer score in the vehicle control group (2.0 ± 0.6325) as compared to naive. Meth-treated (0.2500 ± 0.4183; *P* < 0.001), EA-treated (0.6667 ± 0.8165; *P* < 0.01), and NH-treated (0.3333 ± 0.5164; *P* < 0.001) groups showed reduction in ulcer score as compared to the vehicle control group. Similarly, omeprazole treatment (0.3333 ± 0.4082; *P* < 0.001) also caused suppression of ulcer score as compared to the vehicle control group (Figure 4).

### 3.5. Effects of *P. reticulatus* on IL-8 mRNA Expression Levels

Results showed elevated (*P* < 0.001) mRNA expression levels of IL-8 in the vehicle control group as compared to naive (2.733 ± 0.8029 vs. 1 ± 0.4102). Meth-treated (1.308 ± 0.7010; *P* < 0.01), EA-treated (1.172 ± 0.4001; *P* < 0.01), and NH-treated (1.706 ± 0.4913; *P* < 0.05) groups showed significant downregulation in IL-8 levels as compared to the diseased group. Similarly, omeprazole treatment (1.369 ± 0.4177; *P* < 0.01) also caused downregulation of IL-8 levels as compared to the vehicle control group (Figure 5(a)).

The article "Phyllanthus reticulatus Prevents Ethanol-Induced Gastric Ulcer via Downregulation of IL-8 and TNF-α Levels" was published in 2021. Journal: Evid Based Complement Alternat Med.

### 3.6. Effects of *P*. *reticulatus* on TNF-*α* mRNA Expression Levels

The data demonstrated upregulation (*P* < 0.01) in the levels of TNF-*α* in the vehicle control group as compared to naive (2.291 ± 0.6945 vs. 1 ± 0.5749). Meth-treated (1.237 ± 0.4829), EA-treated (1.409 ± 0.4912), and NH-treated (1.277 ± 0.5750) groups showed reduction (*P* < 0.05) in the mRNA expression levels of TNF-*α*. Similarly, omeprazole treatment also downregulated TNF-*α* levels (*P* < 0.05) compared to the vehicle control group (1.171 ± 0.1882) (Figure 5(b)).

## 4. Discussion

Gastrointestinal ulcer is a disease that mainly occurs in the inner layer of the stomach lining or near the duodenum [20]. Gastric ulcer is one of the most common disorders, and a significant number of people are affected with this disease around the world. The development of gastric ulcers is a complex and multifactorial pathological condition that affects a balance between aggressive and preventive factors present in the gastric mucosa [21]. Increased incidence of gastric ulcers is associated with aggressive factors against the gastric mucosa such as ethanol exposure, stress, smoking, nutritional deficiencies, hereditary predisposition, infection by *Helicobacter pylori*, and frequent ingestion of nonsteroidal anti-inflammatory drugs [22]. Major key factor causing gastric ulcer is the presence of high gastric acidity which can potentiate the action of aggressive agents within stomach mucosa [23]. Pathogenesis of gastric ulcer involves infiltration of inflammatory cell with poly morpho nuclear (PMN) neutrophils, lymphocytes, and eosinophils [24].

Medicinal treatment derived by plants is common and extends to traditional and modern medicinal practice. *Phyllanthus reticulatus* has been used in traditional Asian medicine for the treatment of diseases such as inflammation, diabetes, and microbial infections and as analgesic and hepatoprotective [25]. In the current study, we used the ethanol-induced gastroulcer rat model to analyze the antiulcer and immunomodulatory activities of *Phyllanthus reticulatus* as this model resembles human acute gastric ulcer [26]. It is the most commonly used model to induce gastric ulcer because this method is rapid and is an easy way to evaluate antiulcer activity of plant extract or active ingredient [13]. Ethanol causes direct and indirect damage to the stomach. Direct injury is caused with rapid entry into stomach lining, resulting in vascular endothelial dysfunction. This effect is attributed to hypoxia, hemorrhagic necrosis, and reduction in gastric mucus secretion. As a result, the flow of Na^+^/K^+^ and secretion of pepsin increases, and H^+^ accumulates in the gastric cavity [13, 27]. The indirect damage is ascribed to the recruitment of leukocytes that stimulates the inflammatory responses by increasing the levels of various proinflammatory cytokines [28]. A significant elevation in the total ulcer score, reduction in pH value, and rise in gastric acidity was determined in the ethanol only administered group. These changes of gastric mucosal inflammation are consistent with the studies previously performed [29, 30]. Pretreatment with plant extracts significantly inhibited all these ethanol-induced gastric effects. These results are comparable with the inferences of previous studies [31, 32].

The article "Phyllanthus reticulatus Prevents Ethanol-Induced Gastric Ulcer via Downregulation of IL-8 and TNF-α Levels" was published in 2021. Journal: Evid Based Complement Alternat Med.

*P. reticulatus* extracts significantly reduced the severity of erosion score, hemorrhage score, fibrinoid necrosis score, inflammatory infiltrate score, edema score, and ulcer score. Rats that received pretreatment with *P. reticulatus* had comparatively better protection of the gastric mucosa as observed by marked reduction of different parameters. The research studies previously done showed that TNF-*α* and IL-8 play an important role in causing gastric mucosal lesions as their levels are significantly increased in ethanol-induced stomach ulcer [33, 34].

Proinflammatory cytokine TNF-*α* has pleiotropic roles [35]. It plays crucial role in the formation of gastric ulcer by eliciting an acute inflammatory reaction accompanied by neutrophil infiltration in gastric mucosa [36]. It also regulates apoptotic cell death in the gastric mucosa [36, 37]. It is known to suppress gastric microcirculation, cell proliferation, and angiogenesis at the ulcer margin, thus delaying ulcer healing [28, 38]. Therefore, it may be perceived that reduction in the TNF-*α* level might facilitate ulcer healing. In this context, TNF-*α* expression levels were examined in our study, and results revealed elevated levels in the positive control group which were found significantly attenuated in *p. reticulatus* treated groups. Our findings are in line with the results of Du et al. and Jainu et al. [39, 40]. These studies suggested that the amelioration of stomach ulcer with *Veronicastrum axillare* and *Cissus quadrangularis* extracts was attributed to the reduction in the raised TNF-*α* levels.

IL-8 is an important chemotactic and activating factor for neutrophils. The secretion of IL-8 by epithelial cells is probably a key factor in host defences at mucosal sites, permitting a rapid polymorph response against infectious agents. If defence mechanisms fail and chronic infection results, continued upregulation of IL-8 and neutrophil activation could lead to mucosal damage and increased free radical formation. Mucosal IL-8 production and *H. pylori* infection are two important factors in the immune-pathogenesis of peptic ulcer disease and may also be of relevance to gastric carcinogenesis [41, 42]. IL-8 is a multifunctional inflammatory cytokine that is considered a major controller of acute and chronic-inflammation. Earlier studies revealed that mRNA expression levels of IL-8 were significantly increased in gastric stomach ulcer [21, 43]. We determined the effects of extracts of *P. reticulatus* on mRNA expression levels of IL-8 and found significant reduction in the treated groups as compared to the diseased group.

The article "Phyllanthus reticulatus Prevents Ethanol-Induced Gastric Ulcer via Downregulation of IL-8 and TNF-α Levels" was published in 2021. Journal: Evid Based Complement Alternat Med.

Our findings are in line with the results of earlier studies which attributed the gastroprotective effects against pylorus ligature-induced gastric ulcer in rats to reduce the raised IL-8 levels [44].

## 5. Conclusion

Current research proposes that *P. reticulatus* possesses substantial antiulcer property which might be ascribed to anti-inflammatory and immunomodulatory activities. The data showed significant reduction in ulcer score, erosions, edema, hemorrhage, fibrinoid necrosis, inflammatory cell infiltration, and gastric acidity. These results might be attributed to downregulation of IL-8 and TNF-*α* levels. To what extent, *P. reticulatus* clinically changed the intensity of inflammatory and immunomodulatory cytokines need more research studies.

## Figures and Tables

**Figure 1:** Gastric mucosa of animal from the naive control group showing normal architecture and structure. Mucosal glands showing normal ductal structure (a). Gastric mucosa of rats from the vehicle control group showing infiltration of inflammatory cells, erosions, and ulcer (green), sloughing of epithelial cells (blue), and also extensive fibrinoid necrotic areas with edematous transudate (yellow) (b). Gastric mucosa of rats from the Meth-treated group showing mild inflammatory infiltrate score and edematous mucosa (green). It shows no hemorrhage. Mild epithelial erosion is visible (yellow). Extensive fibronecrotic change was present (c). Gastric mucosa of rat from the NH-treated group showing no hemorrhage score. It shows mild fibrinous necrosis and edema (red). It shows multifocal sloughing of epithelial cells and disarray of the epithelial lining (green) (d). Gastric mucosa of animals from the EA-treated group showing no inflammatory cells, no hemorrhage, and ulcer. High columnar epithelia and normal architecture of mucosal glands is also detected (green) (e). Gastric mucosa of rat from the OM-treated group showing mild erosion (green) and no hemorrhage. It shows edematous mucosa (red) and no inflammatory infiltrate score (f).

The article "Phyllanthus reticulatus Prevents Ethanol-Induced Gastric Ulcer via Downregulation of IL-8 and TNF-α Levels" was published in 2021. Journal: Evid Based Complement Alternat Med.

**Figure 2:** The pH values were found significantly increased in all treated groups compared to the vehicle control group (*P* < 0.001).

**Figure 3:** The total acid secretin was substantially decreased (*P* < 0.001) in all treated groups as compared to the vehicle control group.

**Figure 4:** All treatment groups showed reduction in the ulcer score as compared to the vehicle control group. The data were analyzed using the Kruskal–Wallis test followed by Dunn's multiple comparison test.

**Figure 5:** The data showing P. *reticulatus* significantly reduced the mRNA expression levels of IL-8 (a) and TNF-*α* (b) as compared to the vehicle control group.

**Table 1:** Histopathological scoring of gastric mucosa of rats.

Groups	Erosion score	Ulcer score	Hemorrhage score	Fibrinoid score	Inflammatory infiltrate score	Edema score
Naïve	0	0	0	0	0	0
Vehicle control	5	5	2	4	4	5
Meth-treated	2	3	0	4	2	2
NH-treated	1	3	0	2	3	2
EA-treated	0	1	0	3	1	2
OM-treated	1	2	0	1	0	3

## Data Availability

The data used to support the findings of this study are available from the corresponding author upon request.
